This article has been retracted.

# A study on the strength and durability characteristics of fiber-reinforced recycled aggregate concrete modified with supplementary cementitious material

**DOI:** 10.1016/j.heliyon.2023.e19978

**Published:** 2023-09-09

**Authors:** Osama Zaid, Fadi Althoey, Rebeca Martínez García, Jesús de Prado-Gil, Saleh Alsulamy, Mohammed Awad Abuhussain

**Affiliations:** a Department of Civil Engineering, Swedish College of Engineering and Technology, 47070, Wah Cantt, Punjab, Pakistan; b Department of Civil Engineering, College of Engineering, Najran University, Najran, Saudi Arabia; c Department of Mining Technology, Topography, and Structures, University of León, Campus of Vegazana S/n, 24071, León, Spain; d Department of Architecture and Planning, College of Engineering, King Khalid University, Abha, 61421, Saudi Arabia; e Architectural Engineering Department, College of Engineering, Najran University, Saudi Arabia

**Keywords:** Mechanical strength, Durability performance, Polypropylene fibers, Recycled aggregate, Wheat straw ash

## Abstract

Recycled aggregate (RA) made from waste concrete is an environmentally friendly alternative to natural aggregate (NA) for concrete manufacturing. However, compared to NA concrete, concrete produced with recycled aggregates has poor characteristics. Supplementary cementitious materials (SCMs) can be used to enhance the poor properties of recycled aggregate concrete (RAC). Silica fume and fly ash are commonly used SCMs in the World, but their high usage led to a shortage of silica fume and fly ash. Still, the deficiency of these materials in large parts of the world is a challenge that requires exploring alternative feedstock materials for the construction industry in the coming years. Wheat straw ash (WSA) is an agricultural waste product that could be used as an alternative SCM due to its pozzolanic behavior to enhance the properties of RAC. In addition, concrete is brittle and needs reinforcement, for which polypropylene fibers (PPFs) can be used. The current research examines the mechanical characteristics of fiber-reinforced RAC, including compressive strength, splitting tensile strength, and ductility performance. Durability indicators, such as chloride diffusion, chloride penetration, acid resistance, and water absorption test, were also assessed. The results showed that concrete samples with 10% WSA, 50% RA and 1.5% PPFs had the highest compressive and splitting tensile strength, 60.2 MPa and 7.25 MPa, respectively, representing increases of 24.75% and 30.65%, as compared to plain samples at 56 days. In these samples, water absorption was reduced by 13% due to the finer WSA particles resulting in the lowest reduction in strength and mass recorded when exposing concrete samples to acidic media. The statistical analysis also validated that irrespective of WSA and PPFs, the concrete with 0% RA had the highest performance in strength and durability behavior. The study showed that WSA and PPFs might be employed in tandem to offset the poor behavior of RA, enhance the bond between fibers and concrete, and improve the mechanical strength and durability performance of RAC, thus demonstrating its suitability as a sustainable and economical construction material.

## 1 Introduction

In recent years cement production has quickly grown [1] due to significant increases in housing needs and demand for infrastructure development [2]. Fulfilling this considerable interest requires an enormous cement supply [3]. In 2018, cement production exceeded 4111.1 million tons [4], the most consumed material next to water [5]. Manufacturing cement is an energy-consuming procedure that accounts for approximately 5% of worldwide carbon dioxide (CO_2_) emissions [6]. In addition, increases in cement demand anticipate further increases up to 8% [7], which is huge for a single industry. Increasing cement replacement by supplementary cementitious materials (SCMs) up to 25% has been identified as a promising strategy to reduce the ascent release of CO_2_ in construction-related activities [8,9]. Besides, new urbanization and rehabilitation projects form a large volume of concrete waste around the globe, and when demolished concrete debris is dumped in landfills, it causes serious environmental issues [10]. Alternatively, this waste stream can be upcycled into useful construction materials by utilizing it as alternative aggregates in concrete manufacturing [11]. Recycled aggregates can be obtained by removing waste concrete from construction [12,13] and demolition waste, crushing, sieving, and cleaning the produced aggregates to remove fine particles and impurities [[12], [13], [14]].

Similar to partially replacing cement with SCMs [15], using recycled aggregates leads to a reduced request for natural aggregates [16], which can help lessen the detrimental environmental impacts of construction. In addition, some recent studies have shown that CO_2_ curing can further improve the ecological profile of recycled concrete aggregates [[17], [18], [19]]. Generally, recycled aggregates comprise 65%–80% of natural aggregates and 35%–20% of adhered old cement binder paste [20]. The mechanical properties and other attributes of recycled concrete aggregates are impacted by the parent concrete source attributes, such as proportioning of mixes and workability [21]. The durability and mechanical characteristics of concrete samples produced with recycled concrete aggregates are generally worst as related to equivalent samples produced with limestone or granite aggregates [22]. The high porosity of recycled aggregates and weak interfacial zones amid new and aged concrete has been suggested as the possible causes for RCA's detrimental effects on concrete characteristics [23,24]. Another central concern is the long-term durability of recycled aggregates in concrete [25]. However, the harmful effects of recycled concrete aggregates might be controlled using mineralogical admixtures and pozzolanic materials as cement substitutes [[26], [27], [28]]. These additives contribute to filling the porous microstructure of recycled concrete aggregates with calcium silica hydrate gel (*C*–S–H), thereby densifying the structure of RAC [29], ultimately improving its mechanical performance and durability [30]. Silica fume, fly ash, and other natural and manufactured materials can be used as pozzolans to enhance concrete performance [31]. However, regional shortage of SCM may affect limited concrete upcycling rates [32]. The enforcement of stringent environmental restrictions is expected to exacerbate further existing deficiencies of some SCMs [33] (e.g., see the case of the State of Miami, USA, where the promotion of alternative energy sources has caused massive deficiencies in fly ash availability [34].

Consequently, traditional pozzolan resources are short in supply. There is an urgent need to explore alternative eco-friendly SCMs [35] that could alleviate RA's inferior behavior to enable higher valorization rates of concrete waste [36]. Wheat straw ash is one of the recent interesting materials in the scientific community as supplementary cementitious materials [37]. Wheat straw ash (WSA) is a cereal production waste product; farmers burn wheat straws in open fields [38]. When wheat straw is burned in a controlled environment, a SiO_2_-rich ash is formed with pozzolanic characteristics that can be used as supplementary material in concrete [39]. Using WSA will have several benefits, including reducing CO_2_ emissions in the atmosphere by lowering the clinker factor in concrete, a cost-effective solution to the construction industry, and positive technical effects on concrete properties [40]. As SCMs, fibers can also develop cement-based materials with improved mechanical and durability characteristics [41,42]. The fiber dosage and type significantly affect the concrete properties [43]. Polypropylene fibers (PPFs) are one of the most used reinforcement materials in the construction industry [[44], [45], [46]]. Fiber-reinforced concrete is primarily used to deliver improved impact resistance, ductility, and toughness [47]. Concrete tensile and durability can also be enhanced with PPFs fibers [48]. In addition, PPFs have been shown to restrain microcracks development and decrease microcrack spread in concrete [49,50]. Hanumesh et al., 2018 [51] utilized PPFs in RAC and noticed increases in shear strength and mechanical characteristics with 25% recycled aggregate [52]. The authors suggested permissible limits of 1% PPFs and 50% RA [53]. The impact of utilizing different PPFs dosages in concrete produced with natural aggregate [54] and 100% recycled concrete was previously examined [54,55]. Das et al. [55] observed that the ideal content of PPFs was 0.7%, and the impact of PPFs on tensile strength was more significant compared to compressive strength, thus revealing to be a very suitable material to improve the brittleness of concrete [56].

Many experimental investigations have studied the unique individual benefits of adding mineral admixtures, SCMs, or fibers in recycled aggregate concrete. To the authors' best information, no significant research has been performed on combining polypropylene fibers with wheat straw ash as a partial substitute for cement in recycled aggregate concrete to evaluate the strength and durability properties of concrete which signifies the novelty of the present research. Compressive strength, split tensile strength, and ductility tests were conducted for mechanical tests. Chloride ion diffusion, chloride penetration, water absorption, strength, and mass loss due to acid resistance tests were investigated for durability assessment. Lastly, statistical analysis was performed to validate the lab results. The present study will help readers develop information about improving the properties of recycled aggregate concrete modified with wheat straw ash and polypropylene fibers. The present study will assist in growing awareness of using waste materials (WSA, recycled aggregates) to improve the properties and sustainability of fiber-reinforced concrete.

## 2 Materials and methods

### 2.1 Materials

#### 2.1.1 Cement and wheat straw ash

The present research used Type I cement per ASTM C150 [57]. WSA can be employed as a pozzolanic material per ASTM C311 [58]. The representative image of WSA is shown in Fig. 1 (a). The physical and mineralogical properties of WSA significantly rely on burning conditions. Especially the burning time and temperature affect the crystallinity and microstructure of WSA [39]. A traditional kiln was used in the present study to burn the wheat straw, replicating field conditions where significant volumes of WSA are produced (Fig. 1 (b)). An electrical device regulated temperature and kept a constant heat rate of 6 ^°^C/min. Wheat straw ash was kept at 600^o^C–800 °C for 5 h. The particle shape and surface texture of WSA are flat and rough, with porosity values above 45% [39]. Wheat straw ash's strength activity index (SAI) was 106.5% per ASTM C618 [59]. X-ray diffraction analysis (XRD) was used to evaluate the crystallinity of wheat straw ash, as presented in Fig. 2. Cement and WSA physical and chemical properties are provided in Table 1. The specific surface of the OPC and WSA was evaluated by utilizing the Blain apparatus per EN 196–6 [60]. Furthermore, BET-specific surface was assessed employing a sorption analyzer (Backman Coulter).

**Fig. 1:** Powdered wheat straw ash (a) and traditional kiln used for burning wheat straw (b).

**Fig. 2:** XRD analysis of wheat straw ash.

**Table 1:** Physical and chemical properties of Ordinary Portland cement (OPC) and wheat straw ash (WSA).

Physical properties		Size	Initial Setting time		Final Setting Time			Soundness		Consistency		Specific surface (cm^2^/kg)	
	OPC	≤75 μm	34 min		410 min			1.70%		32.0%		1664	
	WSA	≤75 μm	–		–			–		–		3230	
Chemical Composition		LOI	SiO_2_	Al_2_O_3_		CaO	Fe_2_O_3_		MgO		SO_3_	K_2_O	Na_2_O
	OPC	2.30	21.40	4.40		61.70	2.30		3.00		2.10	1.70	1.10
	WSA	4.50	48.50	23.00		12.60	5.50		2.50		0.74	3.11	0.05

*LOI: Loss of ignition.

#### 2.1.2 Fine and coarse aggregate

River sand was used as a fine aggregate with a fineness modulus of 2.7, and crushed stone was utilized as a coarse aggregate. A local crusher plant provided RA. Because of RA's high-water absorption, they were saturated before blending in the concrete mix. Fine and coarse aggregates were used in saturated surface conditions. Natural and recycled aggregate details are presented in Table 2, while particle size distribution curves for fine and coarse aggregates are provided in Fig. 3 (a) and (b), respectively. ASTM C 127 [61] and ASTM C 128 [62] were followed to evaluate the specific gravity of coarse and fine aggregates.

**Table 2:** Physical characteristics of fine and coarse aggregates.

Physical Properties	Fine Aggregates	Coarse Aggregates	Recycled Coarse Aggregates (RCA)
Abrasion Resistance (%)	–	21.5	39.7
Fineness Modulus	2.70	4.43	5.10
Absorption Capacity (%)	4.10	2.85	4.65
Specific Gravity	2.66	2.84	2.76
Bulk Density (kg/m^3^)	1566	1575	1489

**Fig. 3:** Particle size distribution of (a) fine sand aggregates and (b) coarse crushed stone (CA) and recycled concrete aggregates (RCA).

#### 2.1.3 Polypropylene fibers

Synthetic polypropylene fibers were used as reinforcement material in concrete production. Polypropylene fibers (PPFs) were purchased from Rawalpindi, Pakistan. PPFs are shown in Fig. 4, and their physical characteristics are displayed in Table 3.

**Fig. 4:** Polypropylene fibers structure.

**Table 3:** Physical characteristics of polypropylene fibers (PPFs).

Physical Properties	Result
Color	White
Length	15 mm
Tensile Strength	650–750 MPa
Breaking Elongation	26%
Density	1.2 g/cm^3^
Young's Modulus	4.5 GPa

#### 2.1.4 Admixture

Third-generation polycarboxylate-based superplasticizer for concrete utilized as a high-range water-reducing admixture as per ASTM C494 [63] to increase concrete workability and flowability. The admixture was added to concrete in all mixtures at a constant proportion of 2% (by binder's weight).

### 2.2 Mixing proportion

Twelve mixes were prepared with gradual increases in recycled aggregate dosage (RA) (0%, 50%, and 100%) in place of natural coarse aggregates (NA). Wheat straw ash (WSA) was used as a cement substitute at a ratio of 10%. The cement replacement level was established based on preliminary laboratory trials and extant literature, which suggest optimal replacement levels in the range of 10% when using recycled aggregates [6]. Moreover, 1.5% of polypropylene fibers (PPFs) by binder's weight were incorporated into the mixes, as shown in Table 4.

**Table 4:** Experimental plan: concrete samples mix design.

Mix ID	Cement	WSA	RCA (%)	PPFs (kg/m^3^)	Coarse Aggr. (kg/m^3^)		Sand (kg/m^3^)	Water (kg/m^3^)	Admixture (kg/m^3^)
					NA	RCA			
WSA-0-No Fiber	550	0	0	0	900	0	880	180	11
WSA-10-No Fiber	495	55		0	900	0	880	180	11
WSA-0-PP Fiber	550	0		8.25	900	0	880	180	11
WSA-10-PP Fiber	495	55		8.25	900	0	880	180	11
WSA-0-No Fiber	550	0	50	0	450	450	880	180	11
WSA-10-No Fiber	495	55		0	450	450	880	180	11
WSA-0-PP Fiber	550	0		8.25	450	450	880	180	11
WSA-10-PP Fiber	495	55		8.25	450	450	880	180	11
WSA-0-No Fiber	550	0	100	0	0	900	880	180	11
WSA-10-No Fiber	495	55		0	0	900	880	180	11
WSA-0-PP Fiber	550	0		8.25	0	900	880	180	11
WSA-10-PP Fiber	495	55		8.25	0	900	880	180	11

### 2.3 Concrete mixing procedure

Wheat straw ash (WSA), fine aggregate, coarse aggregate (RA and NA), and cement were mixed in dry form using a mechanical mixer at an average mixing speed of 70 rpm for 120 s. Then, 60% of the mixing water was added and blended for 70 s. Afterward, PPFs were introduced to the mixture and blended for three more minutes. The remaining water and admixture were added to the blend later and mixed at a speed of 100 rpm for additional 60 s. The concrete blend was left to rest for 30 s, then blending continued for 60 s before fresh concrete tests. Concrete samples were cast and removed from the mold after 24 h of curing and placed in a water tank at 22 °C until their curing was completed. As per ASTM C511-13 [64]. Calcium hydroxide (hydrated lime) was added to the water to prevent the leaching of minerals from the concrete samples. Three specimens were prepared for each concrete mix and trial, and average results were taken as a final value.

### 2.4 Characterization methods

A compression testing machine (CTM) was used for the mechanical testing of cylindrical concrete specimens of 150 mm × 300 mm (diameter x height) as per ASTM C 39 [65]. The compressive tests were performed at 28, 56, and 90 days of curing. Concrete splitting tensile strength test was performed on all 12 concrete mixes samples following ASTM C496 [66] at 28 and 56 days, as detailed in Ref. [67]. A universal testing machine (UTM) was adopted for the stress-strain test. The load was applied to concrete samples in compression, and its stress was evaluated with its corresponding strains for all concrete samples.

A chloride bulk diffusion test was performed on samples after 28 days of curing. After chloride exposure, the samples were cut with an electrical saw machine to determine the diffusion of chloride ions. The outer 100 mm portion of the sample was utilized for testing. Concrete specimens were exposed to 17% (by weight) sodium chloride solution for two months. Sodium chloride solution was procured from an Islamabad chemical factory in a ready-to-use form. Sodium chloride was employed as a high concentration of chlorides in chloride diffusion testing [68]. Equation (1) was used to evaluate the diffusion coefficient in chloride ions following ASTM C1556 [69].

(1) $$C\;\left(x,t\right)=C-\left(C-Ci\right)*erfn\;\left(\frac{x}{\sqrt{4dt}}\right)$$

where C is the surface chloride, C (*x, t*) is the concentration of chloride content at the time (sec) and depth (meters), t is time (sec), C*i* is the primary chloride, *erfn* is the error function, and D is the coefficient of chloride diffusion (m^2^/sec).

For concrete water absorption, ASTM C 1585 [70] was followed, and equation (2) was used to calculate the water absorption of the concrete samples.

(2) $$\text{Water}\;\text{absorption}=\frac{\left(Wsd-Wdry\right)}{Wdry}*100$$

W_dry_ is the specimen oven-dried mass, while W_sd_ is the specimen surface-dried mass after submerging in water.

The resistance of concrete against acid test is demonstrated in terms of loss in mass and reduction in strength after exposing concrete samples to strong acid for a specific period of time. In the current study, a 10% hydrochloric acid (HCl) was employed to evaluate the concrete samples' resistance against acidic media. The test specimens were water cured for 28 days at ambient room temperature, followed by immersion in a 10% solution of HCl acid. To confirm a uniform condition, the specimen's pH was frequently inspected. The test specimens remained in acid for three months and were tested for compression strength afterward. To consider the effect of acid on the concrete's decomposition and strength, loss in mass and reduction in compressive strength of concrete samples were evaluated.

For penetration of the chloride test, concrete samples with 100 mm × 50 mm (diameter x thickness) were used. The samples were cured in water for 28 days and placed in a sodium chloride solution, and when the samples were removed from the test setup, they were sprayed with 0.2 N silver nitrate on the cut piece. The silver nitrate chemically reacts with penetrated sodium chloride to create a compound of white color (silver chloride). The test setup for the chloride penetration is presented in Fig. 5. The penetration of chloride was evaluated in terms of depth (mm).

**Fig. 5:** Setup for the chloride penetration test.

## 3 Results and discussion

### 3.1 Compressive strength

The influence of RA, PPFs and WSA on concrete compressive strength is presented at each curing age in Fig. 6 (a). RA was used to substitute coarse crushed stone at three levels, 0%, 50%, and 100%. At each replacement level and curing age, the most notable strength was observed in blends having both WSA and PPFs, followed by blends with 10% WSA but without PP fibers. Concrete blends with only PP fibers and no WSA presented minor compressive strength improvements. The lowest compressive strength values were observed in reference specimens with no WSA and PP fibers. Nevertheless, the compressive strength of the concrete specimens improved as they aged in all formulations. For 50% recycled aggregates at 56 days, the compressive strength of the modified sample was enhanced by 10.0% and 12.5% with (0% WSA with PP fibers) and (10% WSA with PP fibers) substitution compared to 28 days of strength. After 90 days, for concrete formulations with 50% recycled aggregates, enhancement in strength was 17% and 24% for 0% and 10% cement substitution by WSA, respectively. Compressive strength increased when 10% WSA was incorporated compared to control samples with 0% WSA for fiber and non-fiber reinforced concrete at 28, 56, and 90 days of curing age. It was observed that WSA increased strength development at later ages. This may be attributed to higher hydration rates promoted by the released captivated water in WSA and participation of amorphous silica present in WSA composition [71] to nearby binder matrix as the age of the samples. Also, the rate of strength gaining is greater in fiber-reinforced samples, most likely due to the improved bond created between PPFs and new phases formed due to WSA addition.

**Fig. 6:** (a) Compressive strength of cylindrical concrete specimens produced with different dosages for recycled aggregates Fig. 6 (b) Statistical Analysis for compressive strength of concrete.

#### 3.1.1 Effect of WSA and PPFs on the compressive strength of recycled aggregate concrete

For blends with no WSA, the increase in strength for blends with PPFs is somewhat higher. The difference is considerable for blends having 10% WSA. This is because WSA provides better interaction between PPFs, leading to higher load capacity [43]. Adding WSA enhances the concrete compressive strength. For 10% WSA at 100% recycled aggregates, increases of 5.2%, 6.3%, and 9.6% strength were observed at 28, 56, and 90 days. This increase may be because of the improved Si–*O*–Si bond in the concrete because of a large quantity of reactive silica, which WSA adds to concrete [72]. WSA could affect the surface area by densifying the matrix, improving (refining) the pores, and decreasing the permeability, which causes enhances compressive strength [73]. Concrete compressive strength reduces as the substitution of normal-weight aggregate with recycled aggregate increases. In 100% substitution with recycled concrete aggregate, a strength reduction of 22.4%–29.1% is noted for (WSA0-PP Fibers to WSA10- PP fibers) compared to concrete with normal weight aggregate in entire tested samples. For 50% substitution of normal weight with recycled aggregate, a strength decreases of 9.2%–11.4% for (WSA0-PP Fibers to WSA10- PP fibers) is observed. The decrease in strength is because of old mortar at the RA surface. There are three kinds of interfacial zones in RA concrete [74]. The first zone is between new binder and aggregate [75], the second zone is amid aged and new binder [34], and the third zone is in RA amid aggregate and aged attached binder [76]. The weakest zone is the latter. A microscopic crack in the third interfacial zone can cause low mechanical strength compared to samples produced with natural aggregate (NA) [77]. Overall, the results suggest that WSA promotes the formation of additional phases, which improves bonding with PPFs, thus fully compensating for weaker ITZs formed. Therefore, the combination of WSA and PPFs allows for the replacement of 50% of natural aggregates with minimal loss in strength development after 90 days (WSA-0 no fiber 63.8 MPa; WSA-10, with PPFs 60.2 MPa).

#### 3.1.2 Statistical analysis of compressive strength

Fig. 6 (b) shows a plot of compressive strength at 28 days for all mixes. Each point shown on the graph represents an average of three values. A simple statistical analysis of the plotted data was also performed, and a linear fit curve (line) was also presented for each data series along with the plot equation. It can be observed from the plots shown in Fig. 6 (b) that the maximum compressive strength was recorded in the case of zero (0%) percent replacement of recycled aggregate followed by fifty (50%) percent replacement and then hundred (100%) percent replacement irrespective of the wheat straw ash addition as well as the presence of fibers. This is because the recycled aggregate has a relatively porous structure, and a higher percentage of water absorption was recorded in that case (discussed in section 4.5).

The empirical relationships between tried variable and the value R-square are presented in every statistical analysis Figure. When the value of the R-square is close to unity (1), it signifies an excellent regression response. In most of the statistical analysis, the value of R-square is more than 80%, which indicates that there is a perfect match among the fibers, WSA and recycled aggregates, and the WSA and PPFs are doing their part to mitigate/avert the inferior performance of recycled aggregates. However, in some cases, the R-square value was low, which could be ascribed to the elastic behavior of PPFs. Independently talking about the mixtures, adding wheat straw ash and fibers simultaneously slightly improves the compressive strength in case all mixes. This may be because wheat straw comparatively improves the microstructure [78], and fibers help in tensile failure (compressive failure occurs when concrete fails in tensile during cylinder testing). Regarding the failure patterns during the control and modified sample compression strength test, see Fig. 7 (a); the cracks across modified samples are spread throughout their length. In contrast, control samples failed from the bottom and central areas, see (Fig. 7 (b)).

**Fig. 7:** The test setup used to establish compressive strength. (a) Modified Concrete (WSA-10%, RA-50% with 1.5% Fibers), (b) Control sample.

### 3.2 Splitting tensile strength

The splitting tensile strength test on representative concrete samples is presented in Fig. 8. Fig. 8 (a) shows that concrete samples with fibers did not fail as the fibers prevented the spread of cracks, while in Fig. 8 (b), the control concrete was split wide open during the loading. The effect of RA substitution on splitting tensile strength at 28 days and 56 days is exhibited in Fig. 9 (a). It's noted that the splitting tensile strength of specimens produced with WSA and PPFs and no RA was enhanced by 7.9% from 28 to 56 days of curing, while for the samples with only PPFs, the increase in splitting tensile strength was less significant (6.2%). As RA content was increased, splitting tensile strength was reduced. In concrete samples with 100% RA, a reduction of 23.5% and 16.7% were noted for fiber and non-fiber reinforced samples compared to control samples (i.e., 0% recycled aggregates). The decline in splitting tensile strength might be due to RA concrete's high-water absorption and permeable mortar on the RA surface. Utilizing 10% WSA into no fibrous concrete impacts splitting tensile strength at 28 and 56 days of age. The reduction in split tensile strength for non-fibrous concrete was 1.9% and 5.1% at 28 and 56 days, respectively. A logarithmic curve was utilized to validate the results statistically. The curve line was observed closer to the points during the correlation analysis. The correlation analysis showed with high accuracy that the splitting tensile strength of concrete with 0% had the highest strength regardless of the addition of WSA and fibers. The statistical analysis also revealed (Fig. 9 b) that WSA and PPFs in recycled aggregate concrete have significantly improved the splitting tensile strength. Still, the splitting strength improved with adding WSA and PPFs. The splitting tensile strength of the present study is in line with results previously reported in past research [79]. Polypropylene fibers considerably enhance concrete's splitting tensile strength at an early age as related to the non-fibrous samples. At 50% recycled aggregate, splitting tensile strength increased by 15.3% and 13.4% for WSA10-PPFs and WSA-PPFs at 56 days compared to non-fibrous and non-WSA concrete.

**Fig. 8:** (a) Modified concrete (WSA-10%, RA-50% with 1.5% PPFs), (b) control concrete.

**Fig. 9:** (a) Splitting tensile strength of concrete samples at 28 and 56 days. Fig. 9 (b) Statistical Analysis for splitting tensile strength of concrete.

### 3.3 Stress-strain test

A universal testing machine was employed for stress-strain tests, and the experimental stress-strain curves of samples with different dosages of polypropylene fibers, recycled aggregates, and wheat straw ash are shown in Fig. 10. Stress-strain tests were conducted by applying a compression load with an unvarying crosshead movement at 4 mm/min. ACI 318–14 [80] indicates that concrete samples should display strain values ranging between 0.003 and 0.0035, confirmed in Fig. 10. However, it can be seen that concrete samples with PPFs had a higher strain when compared with reference specimens. However, all samples failed with increasing displacement at mid-span after high loading. The result shows that plain samples were more brittle than the fiber-reinforced recycled aggregate concrete. These results agree with the findings previously reported on steel [81], banana [82] and palm leaf sheath fibers [83]. When using recycled aggregates, Fig. 9 (a) shows that the sample with 10% WSA, 1.5% PP fibers, and 50% RA had a high compression strength, confirmed by the splitting tensile strength test results. The high peaks of specimens were taken as ultimate deformation when subjected to compressive load. As depicted by the area below the displacement curves, PP fiber-reinforced recycled aggregate concrete's fracture toughness was enhanced by adding PPFs and WSA. Still, the highest values for concrete samples with 50% recycled aggregates were found. There is little effect on split tensile strength of further increases in recycled aggregate content (WS10-RCA100-PP1).

**Fig. 10:** Experimental stress-strain curve for concrete samples produced with different recycled aggregate (RCA), wheat straw ash (WSA), and polypropylene fibers (PP) contents.

### 3.4 Chloride ion diffusion

Fig. 11 (a) shows the chloride ion diffusion results measured for each concrete mix at 56 days. It is noted that with 100% RA, the diffusion coefficient increases between 11.3% and 16.2% for WSA10 – PPFs and WSA10 – No PPFs, respectively, for fiber and non-fiber samples. The lower diffusion coefficient value was obtained when fibers and 10% WSA were added to the concrete mixture, followed by concrete with no fiber but 10% WSA. The third lowest value was observed in fiber-reinforced concrete samples having no WSA substitution and 50% RA. It is considered that WSA meaningfully decreases the diffusion of chloride ions; entire all the mixtures with WSA replacement have a low diffusion coefficient as compared to control concrete. The linear statistical analysis (Fig. 11 b) for chloride diffusion shows that the mixtures with the 100% recycled aggregates had the highest chloride diffusion value irrespective of the addition of the polypropylene fibers and wheat straw ash. The reduced diffusion coefficient of WSA concrete can be attributed to the lower porosity and more refined pore structure formed when introducing WSA into the mix design. The WSA ascribe to form CSH gel [84] in a higher amount which refines concrete pore structure. Chloride ion diffusion becomes more pronounced as substituting RA is increased due to the open nature of structures formed related to porous ITZ between new and aged binders [85]. Nevertheless, if RA content is limited to 50%, minor increases in diffusion can be attained with the simultaneous addition of PPFs and WSA.

**Fig. 11:** (a). Chloride diffusion coefficient of concrete samples produced with different recycled aggregate (RCA), wheat straw ash (WSA), and polypropylene fibers (PP) contents. Fig. 11 (b) Statistical Analysis for chloride diffusion (mm).

### 3.5 Water absorption

Water absorption tests can be used to estimate concrete porosity. Pore connectivity and tortuosity impact the volume of permeable voids in concrete. This testing was conducted on specimens placed in water for 56 days, and the water absorption values of various samples are shown in Fig. 12 (a).

**Fig. 12:** (a). Water absorption values (%) of concrete samples produced with different recycled aggregate (RCA), wheat straw ash (WSA), and polypropylene fibers (PP) contents at 56 days. Fig. 12 (b) Statistical Analysis for Water absorption (%) of concrete.

As RA content is increased from 0% to 100% in fiber and no fiber samples, it enhances water absorption by 44.8% and 33.7%. A rise in water absorption is because of the porous and permeable old mortar present in the recycled concrete aggregate. The cracks inside old mortar allow water to flow in a sample [86]. Adding polypropylene fibers raised the water absorption by 8% compared to specimens with no PP fibers. PP fibers enhance the connectivity between the microstructure and the pores, which causes more water absorption. Utilizing 10%, WSA reduced the water absorption by 12.96%, 7.81%, and 7.5% for 0%, 50% and 100% RA as compared to concrete with no WSA and 0%, 50% and 100% RA, which is also presented in terms of statistical analysis as shown in Fig. 12 (b). Finer particles of WSA were arranged uniformly in the matrix and made it dense; hence concrete having WSA had lesser pores. In terms of porosity improvement, it could be observed that the effect of utilizing WSA was higher on PP fiber concrete than on concrete with no PP fibers. WSA enhances the bond between fiber and concrete by filling pores that connect fibers to concrete [85].

### 3.6 Acid resistance test

Two batches of concrete samples were assembled for the acid test to examine the impact on concrete strength due to acid exposure. One batch of concrete specimens was water-cured, while the second was exposed to acid for 28 days using 5% concentrated hydrochloric acid. Representative images of the sample before and after the acid test are shown in Fig. 13 (a) and (b), whereas effects on the strength reduction and mass loss of concrete due to acid attack are displayed in Fig. 14 (a) and (b). Fig. 14 (a) shows that as the amount of recycled aggregate was increased in concrete samples, the compressive strength of concrete samples was reduced after an acid attack. The sample with 100% RA with no WSA and PPFs had the highest reduction in strength (11.3%) relative to its plain counterparts, and the sample with no RA and PPFs but 10% WSA had the lowest impact (7.3%) on its strength reduction. Still, since the purpose of the present work was to determine the optimal mix which has a sufficient amount of recycled aggregates and also utilizes WSA and PPFs, the sample with 50% RA, 10% WSA, and PPFs had the optimized response against acid attack with only 7.5% reduction in strength after acid attack test. The sample utilizing WSA had a lesser strength reduction and mass loss in contrast to the sample with no WSA substitution, which is also confirmed in Fig. 14 (a and b). WSA enhanced the susceptibility against acid exposure in the whole of concrete mixes. Fig. 15 (a and b) also showed that the concrete with 100% RA had the worst effect when placed in acid, as shown in statistical analysis. This might be because of the residual calcium hydroxide content in the WSA sample, which forms concrete more resistant to acid exposure [87].

**Fig. 13:** Concrete samples (a) before and (b) after the acid resistance test.

**Fig. 14:** Effect of acid attack on concrete: (a) the percentage of strength reduction (%), (b) concrete mass loss (%).

**Fig. 15:** Statistical Analysis for acid attack (a) Strength loss (%), (b) Mass loss (%).

### 3.7 Chloride penetration test

Resistance to chloride attack is among concrete's most critical durability characteristic due to the corrosion of steel reinforcement bars. Hence its measurement is fundamental for engineers' design of concrete structures, especially for coastal and marine environments. Concrete samples were immersed in sodium chloride (NaCl) solution for 28 days to conduct a chloride penetration test. Values obtained from various mixes of chloride penetration tests are shown in Fig. 16. It was observed that PPFs don't significantly impact chloride penetration values. However, WSA seems to have a positive behavior against chloride penetration, as the samples with WSA showed lower chloride penetration values than WSA-free counterparts. The results agree with Althoey, F. and Farnam, Y. 2020 [88], who reported similar observations. From the test results, samples with 100% recycled aggregates, 10% WSA and 1.5% PPFs had higher chloride penetration values (13 mm). In fact, higher water absorption values were also observed for samples with 100% recycled aggregates (Fig. 13), in good agreement with forming more porous concrete structures, more susceptible to chloride penetration. Therefore, using recycled aggregates seems to be detrimental to the durability of concrete structures, albeit to a limited extent.

**Fig. 16:** Chloride Penetration (mm) test results of all concrete mixes.

## 4 Practical implementation of the current study

The mass production of cement and its usage in concrete leads to the outflow of greenhouse gases with significant environmental harm. In addition, advancing the world's infrastructure causes increasing demolition and construction waste production, and dumping this waste stream causes massive land pollution. So, to avoid or avert the above issues, it is necessary to utilize a material that is not a waste/recycled material but also eco-friendly. Therefore, wheat straw ash is an appropriate substitute material that can partially replace cement in concrete manufacturing. Also, recycled coarse aggregates from demolition and construction waste can effectively replace natural stone aggregate. However, to offset the detrimental impacts of recycled coarse aggregate, it is necessary to use some reinforcement to make concrete more ductile. Using wheat straw ash will reduce clinker consumption and the cost/budget of a construction project. Similarly, coarse recycling aggregate will help save the natural reserves of limestone and other mineral resources used as aggregates and help preserve the environment.

## 5 Conclusions

In this research, the combined effect of wheat straw ash (WSA), polypropylene fibers (PPFs), and recycled aggregate (RA) on the concrete mechanical performance and durability characteristics were examined. Following are the conclusions that are obtained from the trial investigation.

1. The substitution of natural aggregates with RA substantially impacts concrete mechanical performance and durability characteristics. As the dosage of RA increases, compressive and split tensile strength reduces, and water absorption and diffusion of chloride ions increase, indicating durability reductions.
2. With 10% WSA, 50% RA and 1% PPFs, the compressive strength was increased up to 24% at 90 days of curing relative to reference samples.
3. At 50% RA level, splitting tensile strength was increased by 15.3% and 13.4% for non-fibrous and non-WSA concrete at 56 days of curing.
4. Including PP fibers improved splitting tensile strength up to 16.6% and 35.6% for 28 and 56 days of curing, respectively.
5. Adding 10%, WSA reduced the water absorption of concrete up to 13.0% due to the finer particles of WSA.
6. The stress-strain curve confirmed the improved ductility behavior of fiber-reinforced concrete, as the sample with 10% WSA, 1% PP fibers, and 50% RA had the highest ductility.
7. With the incorporation of WSA, the durability of RA concrete improves as water absorption is reduced by 13.0%. However, an increasing percentage of RA may lead to less durability because of old mortars present in RA.
8. The simple linear statistical analysis showed that the results presented could be recommended for future studies.
9. WSA addition mitigated RA's inferior durability performance as the lowest reduction in strength and mass due to acid attack was observed when utilizing WSA, RA, and PPFs (7.5% and 5.4%, respectively), which are acceptable values to use concrete in harsh environments.
10. Concrete with 100% RA had high chloride penetration (13 mm), which can lead to detrimental propagation of micro-cracks.
11. PPFs can be used to counteract this adverse effect of RA and improve the cohesion of concrete.

In sum, the results showed that WSA is a potentially viable substitute for cement in concrete manufacturing. WSA enhances mechanical strength and durability performance and improves the performance of fiber-reinforced concrete, most likely due to enhancement in bonds between PP fibers and the concrete binders. Considering the above positive outcomes of the current research, the sustainable fiber-reinforced recycled aggregate concrete developed in the present study deserves further examination related to microstructural analysis (scanning electron microscope, x-ray diffraction, and frontier-transform infrared spectroscopy) as it has demonstrated exciting features to be used in future structural applications.

## Funding

No funding

### Author contribution statement

Osama Zaid, PhD: Performed the experiments; Wrote the paper. Fadi Althoey, PhD; Saleh Alsulamy, PhD: Analyzed and interpreted the data. Rebeca Martínez García, PhD: Conceived and designed the experiments; Wrote the paper. Jesús de Prado-Gil, PhD: Conceived and designed the experiments. Mohammed Awad Abuhussain, PhD: Contributed reagents, materials, analysis tools or data.

## Data availability statement

Data will be made available on request.

## Declaration of competing interest

We wish to confirm that there are no known conflicts of interest associated with this publication and there has been no significant financial support for this work that could have influenced its outcome.
